The article "Protective Effect of Dietary Polysaccharides from Yellow Passion Fruit Peel on DSS-Induced Colitis in Mice" was published in 2022. Journal: Oxid Med Cell Longev.

# Protective Effect of Dietary Polysaccharides from Yellow Passion Fruit Peel on DSS-Induced Colitis in Mice

**DOI:** 10.1155/2022/6298662

**Published:** 2022-10-15

**Authors:** Laryssa Regis Bueno, Bruna da Silva Soley, Kahlile Youssef Abboud, Isabella Wzorek França, Karien Sauruk da Silva, Natalia Mulinari Turin de Oliveira, Juliana Santos Barros, Marcelo Biondaro Gois, Lucimara Mach Côrtes Cordeiro, Daniele Maria-Ferreira

**Affiliations:** ^1^Instituto de Pesquisa Pelé Pequeno Príncipe, Curitiba, 80250-060 PR, Brazil; ^2^Faculdades Pequeno Príncipe, Programa de Pós-graduação em Biotecnologia Aplicada à Saúde da Criança e do Adolescente, Curitiba, 80230-020 PR, Brazil; ^3^Department of Biochemistry and Molecular Biology, Federal University of Paraná, Curitiba, Paraná, Brazil; ^4^Instituto de Ciências da Saúde, Universidade Federal da Bahia and Centro de Ciências da Saúde, Universidade Federal do Recôncavo da Bahia, Santo Antônio de Jesus, BA, Brazil; ^5^Faculdade de Ciências da Saúde, Universidade Federal de Rondonópolis, Rondonópolis, MT, Brazil

## Abstract

Inflammatory bowel disease (IBD) is a complex inflammatory disorder characterized by chronic and spontaneously relapsing inflammation of the gastrointestinal tract. IBD includes two idiopathic disorders: Crohn's disease (CD) and ulcerative colitis (UC). In particular, UC causes inflammation and ulceration of the colon and rectum. There is no cure for UC. The pharmacological treatment is aimed at controlling and/or reducing the inflammatory process and promoting disease remission. The present study investigated the possible protective effects of soluble dietary fiber (SDF) isolated from yellow passion fruit peel in the dextran sulfate sodium- (DSS-) induced colitis model in mice, induced by 5% of DSS. The animals were treated with SDF (10, 30, or 100 mg/kg (po)), and the disease activity index was monitored. Colon tissues were collected, measured, and prepared for oxidative stress, inflammation, and histology analysis. SDF improved body weight loss, colon length, and disease activity index and prevented colonic oxidative stress by regulating GSH levels and SOD activity. Furthermore, SDF reduced colonic MPO activity, TNF-*α*, and IL-1*β* levels and increased IL-10 and IL-6 levels. As observed by histological analysis, SDF treatment preserved the colonic tissue, the mucus barrier, and reduced inflammatory cell infiltration. Although this is a preliminary study, taken together, our data indicate that SDF may improve the course of DSS-UC. More studies are needed to explore and understand how SDF promotes this protection.

## 1. Introduction

Inflammatory bowel disease (IBD) is a general term used to describe chronic inflammatory conditions affecting the gastrointestinal tract, including Crohn's disease (CD) and ulcerative colitis (UC) [1]. IBD is a complex heterogeneous autoimmune disease that presents as a remarkable characteristic of a defect in the protective epithelial intestinal barrier and deregulated immune activation [2]. Although the etiopathogenesis is not fully understood, it is known that IBD stems from an autoimmune background with a strong influence of genetic factors and dysregulated host immunological responses [3], the gut microbiome [3, 4], and exposure to environmental triggers, such as ultraprocessed food intake [5] and psychological stress [6].

The incidence and prevalence of UC have increased worldwide [7], affecting patients of all age groups, particularly between the ages of 15–25 and 50–70 years [7–9]. The clinical presentation of UC includes anemia, weight loss, fever, watery and/or bloody diarrhea, and abdominal pain, which together contribute to an extreme decrease in the patient's quality of life, especially for those with active disease [7, 10]. UC is idiopathic, defined as a chronic, relapsing, and remitting inflammatory disease of the colon, and its diagnosis is based on endoscopic, histological, and laboratory evaluation [7]. The treatment must be adapted to the disease activity (mild, moderate, or severe) and the extent of the colon lesion [11]. Therapies use immunosuppressive and corticosteroid drugs [12], aminosalicylates [13], and monoclonal antibodies, such as anti-TNF-*α* [14] and integrin inhibitors [15]. The main purpose is to induce and maintain remission with the long-term goals of preventing disability, colectomy, and colorectal cancer [16]. However, in addition to the high cost, low efficacy, and side effects, the success of the treatment also depends on several other factors, such as patient adherence and dose optimization [17]. Therefore, various new therapeutic strategies with natural compounds have been studied for UC treatment [18].

Many studies have reported that dietary fibers (nondigestible polysaccharides) ameliorate intestinal barrier function through the improvement of gastrointestinal flora diversity [19–22] and reduction of intestinal barrier defects and inflammation [23]. Our research group has been dedicated to studying the polysaccharides obtained from biomass residues from the yellow passion fruit (*Passiflora edulis* f. *flavicarpa*), an unexplored coproduct of the juice industry. In addition to the already known nutritional value (vitamin B_3_, iron, calcium, and phosphorus) [24], the consumption of passion fruit offers several beneficial therapeutic effects, including antioxidant, anti-inflammatory [25], hypoglycemic, and vasorelaxant [26]. It has also been observed that soluble dietary fibers from passion fruit peel flour presented an antigastric ulcer effect *in vivo* [27]. Therefore, our study is aimed at investigating whether soluble dietary fiber (SDF) from yellow passion fruit peel (*P. edulis f. flavicarpa*) could improve the course of ulcerative colitis induced by DSS in mice, by reducing the inflammatory process and promoting tissue healing.

## 2. Methods

### 2.1. Soluble Dietary Fiber Extraction

Soluble dietary fiber (SDF) was obtained from yellow passion fruit (*Passiflora edulis f. flavicarpa*) peel. Briefly, the fruits were washed, and the peel was separated from the pulp, cut into small pieces, and then dried at 50°C. The dried matter was made into flour and stored at room temperature until analysis as previously described [27]. SDF's relative molecular weight was 53 kDa; it is composed of 92% of GalA with high methyl esterified homogalacturonan [27].

### 2.2. Animals

All experimental protocols were approved by the Animal Use Ethics Committee of the *Instituto de Pesquisa Pelé Pequeno Príncipe* (number 055-2020). All procedures followed the Guide for the Care and Use of Laboratory Animals (8th edition, National Research Council, 2011) and the Brazilian National Council for the Control of Animal Experimentation. Female Swiss mice (20–30 g), aged between 4 and 5 weeks, were provided by the Animal Facility of *Instituto Carlos Chagas*, *Fiocruz*, Curitiba, PR, and kept in plastic cages (maximum 12 animals per cage), covered by a layer of wood shavings. Animals were housed and fed in a controlled environment at a temperature of 25 ± 2°C and a 12 h light/dark cycle and acclimatized for at least 1 week before the experiments. Wood shavings and the environmental enrichment were changed every three days, and the animals were maintained with *ad libitum* access to standard laboratory chow and water. For the ulcerative colitis induction protocol, the animals were randomized, matched for weight, and identified according to their group.

### 2.3. Dextran Sodium Sulfate (DSS) Colitis Model

Acute ulcerative colitis was induced by 5% of DSS (dextran sodium sulfate, molecular weight: 40,000, Cayman Chemical Company), given to animals in drinking water for 5 consecutive days. On days 6 to 8, the DSS was replaced by normal drinking water. The disease's clinical course was monitored daily throughout the experimental protocol period, and weight loss, change in stool consistency, and rectal bleeding were scored (disease activity index (DAI)). On day 8, all animals were euthanized, and the colons were removed, measured, and stored for further analysis.

### 2.4. Pharmacological Treatments and Disease Activity Index (DAI)

The experimental protocol and treatment are illustrated in Figure 1. Mice were divided into the following treatment groups: (i) control group that received only drinking water (control: water, 1 mL/kg (po)); (ii) DSS group, treated with vehicle and given DSS in drinking water (DSS: water, 1 mL/kg (po)); and (iii) SDF group, treated with SDF and given DSS in drinking water (SDF: 10, 30, or 100 mg/kg (po)).

The DAI was monitored daily and scored according to the animal's body weight changes as follows:

- 0: increased or remained within 1% of the baseline
- 1: decreased by 1 to 5%
- 2: decreased by 5 to 10%
- 3: decreased by 10 to 15%
- 4: decreased by more than 15%

The stool consistency was scored as follows:

- 0: in the absence of diarrhea
- 2: if the stool did not stick to the animal's anus
- 4: if the animal presented liquid stool

The presence of blood in stool was scored as follows:

- 0: if animals did not present blood in stool
- 2: for moderate blood in stool
- 4: for gross bleeding

At the end of the experimental protocol, the colon tissues were carefully removed and washed with 0.9% saline. The lengths were measured, and the tissues were stored at -80°C for further analysis.

### 2.5. Tissue Preparation

Animal tissues were homogenized in PBS (pH 7.4) containing protease inhibitor (Sigma FAST™). The homogenate was analyzed for glutathione (GSH) levels. The samples were centrifuged at 8,900 rpm at 4°C for 20 min. The supernatant was used to determine the superoxide dismutase (SOD) activity, cytokines, and protein levels. The pellet was resuspended in phosphate buffer with hexadecyltrimethylammonium (HTAB) and used to measure myeloperoxidase (MPO) activity.

Cytokine levels (TNF-*α*, IL-1*β*, IL-6, and IL-10) were evaluated using an enzyme-linked immunosorbent assay (ELISA) kit according to the manufacturer's recommendations (PeproTech Inc.). The protein concentration was determined by the method of Bradford (Bradford, 1976), using the bovine serum albumin standard curve. All results were read in a spectrophotometer as recommended and interpolated with their respective standard curves.

### 2.6. Determination of GSH Levels and SOD Activity

To determine the GSH levels, 50 *μ*L of tissue homogenate was mixed with 40 *μ*L trichloroacetic acid (12.5%) and vortexed for 10 min. The samples were then centrifuged for 15 min at 3,000 rpm at 4°C, and aliquots of 10 *μ*L of the supernatant were mixed with Tris buffer (400 mM, pH 8.9) and 5,5′-dithiobis (2-nitrobenzoic acid) (DTNB, 10 mM). This solution reacts with GSH to generate a yellow compound (2-nitro-5-thiobenzoic acid). The reaction absorbance was measured using a spectrophotometer at 415 nm. All values were interpolated into a standard curve of GSH (0.375–3 *μ*g), and the results were expressed as *μ*g of GSH per mg of protein [28, 29].

Supernatant aliquots of 20 *μ*L were added to a buffer solution containing 200 mM Tris HCl-EDTA (pH 8.5) and pyrogallol (1 mM) to measure the SOD activity. The samples were vortex for 1 min and incubated for 20 min at room temperature. The reaction was stopped with 1 N HCl. All samples were centrifuged for 4 min at 14,000 rpm. The absorbance was read by a spectrophotometer at 405 nm, and the amount of SOD that inhibited the pyrogallol oxidation by 50% was defined as one unit (U) of SOD activity (relative to the control of the test). The enzymatic activity was expressed as units per milligram of protein (U/mg of protein) [29].

### 2.7. Quantification of MPO Activity

The MPO activity was determined by using the sample pellets. Briefly, the pellets were resuspended in 1 mL of potassium phosphate buffer (80 mM, pH 5.4) containing 0.5% hexadecyltrimethylammonium bromide (HTAB). After, the samples were centrifuged at 9,900 rpm for 20 min at 4°C. Then, 30 *μ*L of the supernatant was mixed with 0.017% of H_2_O_2_ and 3,3′,5,5′-tetramethylbenzidine (TMB, 18.4 mM). The reaction absorbance was measured at 620 nm, with the results expressed as optical density (OD)/mg of protein [30].

### 2.8. Determination of Cytokine Levels

Samples were centrifuged at 8,900 rpm at 4°C for 20 min, and the supernatant was used to measure cytokine levels; the levels of IL-1*β*, TNF-*α*, IL-10, and IL-6 were evaluated using an enzyme-linked immunosorbent assay (ELISA) kit according to the manufacturer's recommendations (PeproTech). Each cytokine level was extrapolated from a standard curve (pg/mL), and the results were expressed as pg of each cytokine/mg of protein.

### 2.9. Histopathological and Immunohistochemical Assessment

Colon samples were collected from the same defined regions, fixed in 10% formalin (neon), and dehydrated sequentially in ethanol and ether for inclusion and construction of paraffin blocks. The paraffin blocks were sectioned in a microtome (7 *μ*m thickness cross-section). Slides containing the histological sections were deparaffinized and stained with hematoxylin and eosin (H&E) for histopathological evaluation. H&E-stained colonic tissue sections were blindly scored by assessing infiltration of the lamina propria with mononuclear cells, crypt hyperplasia, goblet cell depletion, and alteration of mucosal histoarchitecture (including epithelial erosion and mucosal ulceration), resulting in scores of 0 to 6 (Table 1) [31, 32]. Ten microscopic fields from each mouse, from at least 8 mice per group, were examined using a light microscope (Olympus® BX43F, Minato-Ku, Japan) and a 20x objective (and 40x or 100x if necessary to confirm structure). Slides were also stained for periodic acid Schiff (PAS) and Alcian Blue (AB), and stained mucin-like glycoprotein positive pixels were captured and quantified with the ImageJ® software.

For immunohistochemical evaluation of mucin 1 (MUC-1), slides containing the histological sections were deparaffinized, incubated overnight with primary anti-MUC-1 antibodies (1 : 100, pH 9) (rabbit polyclonal to MUC1 IgG, 1 : 100, Abcam), and revealed with 2, 3, diamino-benzidine complex + hydrogen peroxide substrate. Positive pixels were captured and quantified with the ImageJ® software.

### 2.10. Statistical Analysis

The Shapiro-Wilk test was used to assess the normality of the data. Statistical analysis was performed using Kruskal-Wallis, followed by Dunn's posttest for nonparametric data. The results were expressed as a median with interquartile ranges. One-way ANOVA or two-way ANOVA followed by Bonferroni's multiple comparisons posttest for multivariable analyses was applied to compare differences between multiple groups that presented parametric data. The results were expressed as means ± SEM. Differences with *p* < 0.05 were considered statistically significant. All analysis was conducted using the GraphPad Prism software (GraphPad Software).

## 3. Results

### 3.1. SDF Treatment Alleviated DSS-Induced Colitis

The animals were treated orally once a day with SDF (10, 30, and 100 mg/kg) or vehicle (water, 1 mL/kg), from day 1 to day 7 (Figure 1) to assess the potential effect of SDF in the DSS-induced colitis model. The body weight change and DAI were evaluated according to the experimental protocol. At the end of the experiment (day 8), the animals were euthanized; the colons were collected, measured, and stored for further analysis.

The animals that received DSS in drinking water and were treated with vehicle started to lose weight on day 5 (-4.29%, *p* < 0.0017), continuing up to day 8 (-16.53%, *p* < 0.0001) (Figures 2(a) and 2(b)) when compared to healthy mice (control group).

Furthermore, the DSS group presented an increased DAI (days 4, 5, 6, 7, and 8; *p* = 0.0221, *p* < 0.0001, *p* < 0.000, *p* < 0.0001, and *p* < 0.0001, respectively) (Figures 2(c) and 2(d)), as well as a reduced colon length (by 17%), when compared to the control group (median: 9.75 cm) (Figure 3).

The SDF treatment significantly prevented body weight loss (day 8, SDF 30 mg/kg: 86%; day 8, SDF 100 mg/kg: 95%, *p* < 0.0001 and *p* < 0.0001, respectively) (Figures 2(a) and 2(b)) and DAI development (day 8, median SDF 30 mg/kg: 2.5; and day 8, median SDF 100 mg/kg: 1.0, *p* < 0.0001 and *p* < 0.0001, respectively) when compared to the DSS group (median: 8.00) (Figures 2(c) and 2(d)). The treatment with SDF also prevented the reduction in colon length (SDF 30 mg/kg: 12%, *p* < 0.05; and SDF 100 mg/kg: 25%, *p* < 0.001) when compared to the DSS group (median: 8.0 cm) (Figure 3).

The SDF doses of 30 and 100 mg/kg prevented weight loss and the development of DAI when compared to the control group. Therefore, we decided to work only with the highest dose tested (100 mg/kg) in the subsequent experiments, considering that the DSS-induced ulcerative colitis model is a very aggressive inflammatory model.

### 3.2. SDF Decreased Colonic Oxidative Stress

The inflammatory damage induced by DSS brought about the infiltration of neutrophils and macrophages, generating excessive amounts of reactive oxygen species with a subsequent increase in oxidative stress [33]. Therefore, we measured the GSH levels and SOD activity to quantify these parameters.

The animals in the DSS group showed reduced GSH levels (median: 137.1 *μ*g/g of protein) and increased SOD activity (0.53 ± 0.02 U/mg of protein) compared to the control group (median GSH: 218.3 *μ*g/g of protein; median SOD: 0.38 ± 0.00 U/mg of protein) (*p* = 0.0324 and *p* < 0.0001, respectively). The SDF treatment restored the GSH (median: 221.5 *μ*g/g of protein) and SOD activity (0.45 ± 0.01 U/mg of protein) compared to the DSS group (*p* = 0.0129 and *p* = 0.0135, respectively) (Figures 4(a) and 4(b)).

### 3.3. SDF Regulated Colonic MPO Activity and Cytokine Secretion

Colon tissue damage in the DSS-induced ulcerative colitis model is directly linked to increased vascular permeability followed by tissue edema, increased cellular infiltration, such as neutrophils and macrophages, and a consequent increase in mucosal cytokine production [30]. Therefore, we measured colonic pro- and anti-inflammatory cytokines to explore whether SDF treatment could alleviate DSS colitis by regulating inflammation.

We did not observe significant differences in MPO activity between the DSS group (median: 0.20 mg of protein) and the control group (median: 0.15 mg of protein) (*p* = 0.1076). On the other hand, SDF treatment decreased the MPO activity (median: 0.09) (*p* = 0.0101) compared to the DSS group (Figure 5(a)).

An increase in tissue cytokines, including the proinflammatory cytokines IL-1*β* and TNF-*α*, and a decrease in tissue IL-10 and IL-6 were observed in mice that received DSS and were treated with vehicle (IL-1*β*: 5420 ± 583.9 pg/mg of protein; TNF-*α*: 5841 ± 356.5 pg/mg of protein; IL-10: 4217 ± 525.6 pg/mg of protein; IL-6: 2264 ± 265.4 pg/mg of protein), compared to the control group (IL-1*β*: 3598 ± 383.1 pg/mg of protein; TNF-*α*: 2746 ± 520.7 pg/mg of protein; IL-10: 9778 ± 1012 pg/mg of protein; IL-6: 6706 ± 499.2 pg/mg of protein) (*p* < 0.05, *p* < 0.0001, *p* < 0.001, and *p* < 0.0001, respectively). In the SDF group, these cytokines were significantly decreased (IL-1*β*: 3843 ± 248.3 pg/mg of protein and TNF-*α*: 3492 ± 230.5 pg/mg of protein) (*p* < 0.05 and *p* < 0.01, respectively) and increased (IL-10: 7102 ± 877.1 pg/mg of protein and IL-6: 4746 ± 898.8 pg/mg protein) (*p* < 0.05 and *p* < 0.05, respectively) compared to the DSS group (Figures 5(b)–5(e)).

### 3.4. SDF Treatment Improved Microscopic Colon Damage in Mice

Colonic damage induced by oral administration of DSS includes the destruction of the intestinal mucosal barrier and is directly related to the disease progression [33]. Therefore, the colons were collected at the end of the experiment and processed for histological analysis. Then, we further evaluated the protective effect of SDF (100 mg/kg). H&E colon staining (Figure 6) showed that 5% of DSS destroyed the colon tissue, leading to the formation of extensive ulcerations, edema, and histopathological changes in the mucosa and submucosa. SDF (100 mg/kg) H&E-stained sections revealed a significant overall histological improvement, evidenced by a conserved mucosal architecture. Furthermore, the DSS group showed an increase in the histopathological score (median: 4) compared to the control group (median: 2) (*p* < 0.0001). SDF treatment reduced histopathological damage (median: 3) compared to the DSS group (*p* < 0.0001) (Figure 6(a)).

### 3.5. SDF Treatment Preserved the Mucus Layer

A handful of studies have already demonstrated that DSS-induced colonic damage is related to decreased gastric mucus content and secretion [33]. Therefore, we next evaluated if the protective effect of SDF could be associated with the maintenance of the colon's protective mucus barrier. The results show (Figures 7 and 8) that the administration of DSS induced a decrease in PAS and AB staining, indicative of neutral mucin and acid mucin-like glycoproteins (54% and 65%, respectively) (*p* = 0.0016 and *p* < 0.0001, respectively) compared to the control group. The treatment with SDF (100 mg/kg) increased the staining for PAS and AB by 80% and 155%, respectively (*p* = 0.046 and *p* < 0.0005, respectively), compared to the DSS group (34.71 ± 14.51 pixels/field and 2153 ± 613.7 pixels/field, respectively) (Figures 7 and 8).

To confirm the previous result, we performed an immunohistochemical analysis to determine the expression profile of the transmembrane mucin MUC-1. Animals with ulcerative colitis have reduced levels of MUC-1 (95%, *p* < 0.0001) when compared to the control group (Figure 9) (95804 ± 12615 pixels/field). The treatment with SDF (100 mg/kg) increased the labeling for MUC-1 by 300% (*p* = 0.0297) compared to the DSS group (14031 ± 2730 pixels/field) (Figure 9).

## 4. Discussion

Many natural products possess therapeutic and medicinal properties. Bioactive compounds, including polysaccharides formed by polymers of monosaccharides and characterized as macromolecules of high molecular weight, offer various biological activities, such as anti-inflammatory, that could be utilized to develop new IBD therapies [34]. For the first time, we show that the polysaccharides extracted from the yellow passion fruit peel protect mice from ulcerative colitis progression in the DSS model, ameliorate the mucosal barrier, and prevent DSS-induced inflammation.

Inflammatory bowel disease (IBD) consists of two major pathological subtypes: Crohn's disease (CD) and ulcerative colitis (UC) [1]. UC is described as a complex condition becoming increasingly critical globally [35]. The pathophysiology and underlying disease mechanisms remain unclear; however, a handful of studies reported that the disease is directly related to genetic susceptibility, and its occurrence and development have been associated with immune disorders, environmental factors, and mucosal dysfunction [1]. Unfortunately, pharmacological and nonpharmacological strategies for the treatment of UC do not induce cure but aim to reduce symptoms and maintain effective clinical remission [36]. Therefore, the development of safe and effective treatments with a high capacity to maintain the remission of IBD patients is necessary.

There are several experimental models for studying inflammatory bowel disease. The DSS ulcerative colitis model is the most widely used due to its simplicity, high degree of uniformity, and reproducibility of the lesions [37, 38]. Administration of DDS in drinking water induces mucosal damage resulting from the disruption of the intestinal epithelial monolayer lining, luminal bacteria, and associated antigen translocation. Additionally, neutrophils and macrophage infiltration initially mediate oxidative stress and inflammation, contributing to the observed tissue damage [39, 40]. Animals exhibit marked body weight loss, altered stool consistency, and hematochezia [38].

Natural products are gaining ground as possible sources of new options for UC treatment. Several studies have shown that biomolecules have anti-inflammatory activity and can control IBD [18]. Polysaccharides isolated from natural products form one of the main classes of bioactive compounds with therapeutic efficacy [41]. The consumption of nondigestible dietary fibers can provide health benefits and appears to reduce the risk of developing several conditions, including obesity, diabetes mellitus, heart disease, and metabolic syndrome [42, 43]. Interestingly, dietary fibers have also been associated with reducing the risk of developing inflammatory bowel disease, maintaining epithelial barrier integrity, and forming short-chain fatty acids that can inhibit the transcription of proinflammatory mediators [44].

As expected, DSS induced all the characteristics mentioned above in our experiments, including colon shortening. SDF treatment prevented weight loss and increased disease scores, including rectal bleeding, which is directly associated with the prevention of colon shortening [39]. Consequently, all the other aspects of the disease, including raised fur, hunched back, and reduced mobility, were improved. Several other studies have already demonstrated the protective effect of polysaccharides extracted from natural products in ulcerative colitis models [45–47]. Specifically, fruit polysaccharides also have such a protective effect. Zou et al. have demonstrated that *Ficus carica* polysaccharide attenuated DSS-induced ulcerative colitis in C57BL/6 mice by maintaining goblet cells and reducing inflammation [48]. Polysaccharides extracted from *Morinda citrifolia* Linn presented anti-inflammatory action in a mouse acetic acid-induced colitis model, reducing inflammatory cell infiltration and oxidative stress [49]. Related oxidative stress and inflammation were quantified to understand the mechanisms of SDF protection further.

Inflammatory cell infiltration and oxidative stress play an important role in the pathological development, induction, and progression of ulcerative colitis [50]. As the disease progresses, the colonic tissue infiltration of leukocytes, neutrophils, and macrophages increases, resulting in a consequent uncontrolled generation of reactive nitrogen and oxygen metabolites that destroy tissue structures, including lipids, proteins, and DNA [51]. Furthermore, the imbalance between pro- and anti-inflammatory cytokines contributes to compromised immune function and tissue damage [52]. For instance, TNF-*α* derived from dendritic cells, macrophages, and T cells can stimulate the production and release of other proinflammatory cytokines [2]. However, the intestine orchestrates a complex and organized system that contains multiple antioxidant methods of defense and protection mechanisms against inflammation to protect against damage, maintain intestinal integrity, and ensure general and immune homeostasis [53]. We observed in our experiments that SDF treatment prevented oxidative stress by maintaining GSH levels and SOD activity. We also observed that SDF treatment prevented the increase of MPO, TNF-*α*, and IL-1*β* and the reduction of IL-10 and IL-6, suggesting a tissue-protective response and regulatory effect on inflammation. Along with preventing the general development of the disease, it is also possible to suggest that SDF ameliorated colonic inflammation in the DSS-induced ulcerative colitis model.

The inflammatory process observed in the DSS-induced ulcerative colitis model occurs probably due to the intestinal epithelium damage and dissemination of proinflammatory luminal microbial antigens to the underlying tissue [37, 39]. Therefore, reducing the inflammatory process represents an attractive alternative for the management of ulcerative colitis. Interestingly, it has been previously demonstrated that SDF had a protective effect on the stomach mucosa; administering SDF significantly reduced stomach gastric ulcer lesions in rats. The authors also showed that this protection might be related to maintaining GSH levels and gastric mucus secretion, corroborating our data [27]. In addition, it is well-known that the intestinal inflammatory process is directly related to motility dysfunction [54]. We observed through DAI that animals treated with SDF have a lower score of diarrhea when compared to DSS animals. In fact, fiber consumption may modulate gastrointestinal motility either by changes in the microbiota and fermentation end products or by modulating the bulk flow of material through the intestine [55–57]. Moreover, cumulative evidence has shown polysaccharides from different sources and with different structures regulate intestinal motility, reduce diarrhea [58–61], and ameliorate constipation in animals [62–66], adults, and children [67].

Another important factor involved in the pathogenesis of ulcerative colitis is the permeation of the mucous barrier that occurs due to the reduction in the production and secretion of mucins and the stratification of the mucus layers [68]. Mucus barrier abnormalities, such as depleted upper crypt goblet cells, decreased core mucus components, and decreased mucin expression, allow bacterial penetration that could stimulate an abnormal immune system response leading to the development of local tissue inflammation [69]. Tissue inflammation and mucus layer depletion contribute to acute histological changes, which are directly associated with all the colitis aspects, including weight loss and diarrhea [37]. Histological damage, such as modification of normal mucosal histoarchitecture and erosions, and tissue cell infiltration are important changes observed [70, 71]. For this reason, in addition to microscopic analysis, we also assessed mucus preservation through PAS and AB staining and the expression profile of MUC-1. The PAS was employed to stain neutral mucins, and AB was used to stain acid mucin-like glycoproteins in the colon tissue; MUC-1 is transmembrane mucin, and the maintenance of its expression and secretion ensures tissue protection and corrects cell signaling and immune response and consequently intestinal homeostasis [69].

The microscopic examination of the colon sections showed a clear colonic epithelial destruction induced by DSS, with visible tissue damage. We observed a high histological score, which includes cellular infiltration, crypt hyperplasia, epithelial erosion, mucosal ulceration, and goblet cell depletion. The reduction of goblet cells corroborates the results found for PAS and AB staining and MUC-1 expression. It is noteworthy that SDF treatment preserved the epithelial architecture. Histological analyses revealed a reduction in the histopathological score, composed of a reduction in the severity and extent of tissue damage, reduction of erosion, and maintenance of goblet cells. This evidence corroborates the maintenance of positive labeling indicative of mucin. Thus, it is possible to hypothesize that SDF treatment reinforces the protective barrier of the intestinal mucosa, maintaining normal mucus secretion, and thus, intestinal homeostasis.

Cumulative evidence has shown that natural polysaccharides may reinforce the intestinal protective barrier in several ways; furthermore, other studies have shown that these molecules can protect the mucus barrier [72, 73]. Interestingly, chronic or intermittent dietary fiber deficiency can cause erosion of the protective mucus layer, making it thinner and more susceptible to pathogens [74]. Strengthening of the epithelial and mucus barrier can occur, for example, by increased production of short-chain fatty acids (SCFAs) [75]. Increasing the abundance of intestinal *Bifidobacterium*, *Lactobacillus*, and *Escherichia coli* [75, 76] and inhibiting the growth of potentially pathogenic bacteria, such as *Clostridium*, also alleviate ulcerative colitis [77]. Some other authors suggest that polysaccharides reduce the expression of proinflammatory cytokines and MPO activity [76, 78–80].

Finally, we have presented here the protective role of SDF for the first time. However, the exact mechanism by which this polysaccharide extract provides colonic protection is still not entirely clear. Nondigestible polysaccharides have complex structures and may show beneficial properties through direct and indirect mechanisms [81]. The literature assumes that these molecules can, for example, serve as a substrate for bacterial fermentation in the large intestine. This produces SCFAs and other metabolites that interact with different receptors (G-protein-coupled receptors, including GPR41, GPR43, and GPR109A) to promote beneficial effects such as increased prostaglandin production and mucin expression (MUC-1, MUC-2, MUC-3, and MUC-4). Furthermore, it has been shown that polysaccharides extracted from natural products can directly inhibit COX overexpression [82] interact with different mucins through molecular mucoadhesive interactions [83] or interact with Toll-like receptors [84–87].

All these mechanisms could contribute to the observed intestinal protection promoted by SDF. Our results demonstrate that SDF might prevent the development of ulcerative colitis through several mechanisms, including colonic mucosal protection, decreased oxidative stress, and inflammation, ultimately resulting in the maintenance of mucus layer and tissue integrity. Although the exact protection mechanism has not yet been determined, the presented data indicate that SDF may represent an interesting option for managing acute ulcerative colitis. However, more studies are needed to explore and understand how SDF elicits its beneficial effects.

## Figures and Tables

**Figure 1:** Experimental protocol for the induction of ulcerative colitis.

**Figure 2:** Effect of SDF on the (a) body weight change from day 1 to 8, (b) body weight change on day 8, (c) disease activity index from day 1 to 8, and (d) disease activity index on day 8. Animals received 5% of DSS in drinking water for 5 consecutive days followed by 2 days of water. Mice were orally treated, once a day, with vehicle (control or DSS groups: water, 1 mL/kg) or SDF (10, 30, or 100 mg/kg) for 7 days. Results are expressed as mean ± S.E.M. or median with interquartile ranges and analyzed using two-way ANOVA followed by Bonferroni's multiple comparisons test, or Kruskal–Wallis followed by Dunn's, respectively. #*p* < 0.05, compared to control group; ^∗^*p* < 0.05, compared to the DSS group.

**Figure 3:** Effect of SDF on the mouse colon length. Animals received 5% of DSS in drinking water for 5 consecutive days followed by 2 days of water. Mice were orally treated, once a day, with vehicle (control or DSS groups: water, 1 mL/kg) or SDF (10, 30, or 100 mg/kg) for 7 days. Results are expressed as median with interquartile ranges and analyzed using Kruskal–Wallis followed by Dunn's. #*p* < 0.05, compared to the control group; ^∗^*p* < 0.05, compared to the DSS group.

**Figure 4:** Effect of SDF on GSH (a) levels and SOD (b) activity. Animals received 5% of DSS in drinking water for 5 consecutive days followed by 2 days of water. Mice were orally treated, once a day, with vehicle (control or DSS groups: water, 1 mL/kg) or SDF (100 mg/kg) for 7 days. Results are expressed as mean ± S.E.M. or median with interquartile ranges and analyzed using one-or two-way ANOVA followed by Bonferroni's multiple comparisons test, or Kruskal–Wallis followed by Dunn's, respectively. #*p* < 0.05, compared to the control group; ^∗^*p* < 0.05, compared to the DSS group.

**Figure 5:** Effect of SDF on MPO activity (a) and IL-1*β* (b), TNF-*α* (c), IL-10 (d), and IL-6 (e) levels. Animals received 5% of DSS in drinking water for 5 consecutive days followed by 2 days of water. Mice were orally treated, once a day, with vehicle (control or DSS groups: water, 1 mL/kg) or SDF (100 mg/kg) for 7 days. Results are expressed as mean ± S.E.M. or median with interquartile ranges and analyzed using one- or two-way ANOVA followed by Bonferroni's multiple comparisons test, or Kruskal–Wallis followed by Dunn's, respectively. #*p* < 0.05, compared to the control group; ^∗^*p* < 0.05, compared to the DSS group.

**Figure 6:** Effect of SDF on histological parameters and histopathological score (a). Hematoxylin and eosin-stained sections of colons, ×20 (bars = 100 *μ*m). Animals received 5% of DSS in drinking water for 5 consecutive days followed by 2 days of water. Mice were orally treated, once a day, with vehicle (control or DSS groups: water, 1 mL/kg) or SDF (100 mg/kg) for 7 days. Results are expressed as median with interquartile ranges and analyzed using Kruskal–Wallis followed by Dunn's. #*p* < 0.05, compared to the control group; ^∗^*p* < 0.05, compared to the DSS group.

**Figure 7:** Effect of SDF on histochemical staining for neutral mucin-like glycoproteins (PAS) and acid mucin (Alcian Blue). Histochemical staining of colons for neutral mucin-like glycoproteins (PAS) and acid mucin (Alcian Blue), ×20 (bars = 100 *μ*m). Animals received 5% of DSS in drinking water for 5 consecutive days followed by 2 days of water. Mice were orally treated, once a day, with vehicle (control or DSS groups: water, 1 mL/kg) or SDF (100 mg/kg) for 7 days.

**Figure 8:** SDF preserves mucus secretion. Quantification of PAS (a) and Alcian Blue (b). Animals received 5% of DSS in drinking water for 5 consecutive days followed by 2 days of water. Mice were orally treated, once a day, with vehicle (control or DSS groups: water, 1 mL/kg) or SDF (100 mg/kg) for 7 days. Results are expressed as mean ± S.E.M. followed by Bonferroni's multiple comparisons test. #*p* < 0.05, compared to the control group; ^∗^*p* < 0.05, compared to the DSS group.

**Figure 9:** SDF preserves MUC-1 expression. Immunohistochemical staining of colons for MUC-1, ×40 (bars = 500 *μ*m). Quantification of MUC-1 expression (a). Animals received 5% of DSS in drinking water for 5 consecutive days followed by 2 days of water. Mice were orally treated, once a day, with vehicle (control or DSS groups: water, 1 mL/kg) or SDF (100 mg/kg) for 7 days. Results are expressed as mean ± S.E.M. followed by Bonferroni's multiple comparisons test. #*p* < 0.05, compared to the control group; ^∗^*p* < 0.05, compared to the DSS group.

**Table 1:** Histopathological score.

Category	Inflammatory cell infiltrate			Intestinal histoarchitecture		
Criterion	Severity	Extent	Score 1	Epithelial changes	Mucosal histoarchitecture	Score 2
Definition	Mild	Mucosa	1	Focal erosions	—	1
	Moderate	Mucosa and submucosa	2	Erosions	Focal ulcerations, goblet cell depletion	2
	Marked	Transmural	3	Marked erosions	Extended ulcerations ± granulation tissue ± goblet cell depletion	3
Sum of scores 1 and 2						0–6

Score 0: normal.

## Data Availability

The data presented in the current study are available from the corresponding author on reasonable request.
